The article "Effect of Bufalin on Proliferation and Apoptosis of Human Non-small Cell Lung Cancer A549 Cell" was retracted in 2010. Reason: duplicate publication.

# 蟾蜍灵对人非小细胞肺癌A549细胞增殖与凋亡的影响

**DOI:** 10.3779/j.issn.1009-3419.2010.09.01

**Published:** 2010-09-20

**Authors:** 志图 朱, 云龙 郁, 锴 王, 恩泽 李, 阳阳 刘, 云鹏 刘

**Affiliations:** 1 121001 锦州，辽宁医学院附属第一医院肿瘤科 Department of Oncology, the First Affiliated Hospital of Liaoning Medical University, Jinzhou 121001, China; 2 110001 沈阳，中国医科大学附属一院肿瘤内科 Department of Medical Oncology, the First Affiliated Hospital of China Medical University, Shenyang 110001, China

**Keywords:** 蟾蜍灵, 肺肿瘤, 凋亡, Livin, Caspase-3, Bufalin, Lung neoplasms, Apoptosis, Livin protein, Caspase-3 protein

## Abstract

**背景与目的:**

蟾蜍灵是从中药蟾酥中提取出来的有效成分，其抗肿瘤作用已经在许多体外肿瘤细胞中得到证实，本研究旨在探讨蟾蜍灵对人非小细胞肺癌细胞的增殖抑制、诱导凋亡作用及其机制。

**方法:**

采用MTT法测定细胞活力，绘制细胞增殖抑制曲线；瑞氏-吉姆萨染色法观察细胞形态学的变化；流式细胞仪通过PI染色进行细胞周期分析及凋亡判定；Western blot法检测Livin及Caspase-3蛋白的表达。

**结果:**

蟾蜍灵以时间、剂量依赖方式抑制A549细胞增殖，48 h、72 h及96 h抑制细胞增殖50%的药物浓度（half maximal inhibitory concentration, IC_50_）分别为（56.14±6.72）nmol/L、（15.57±4.28）nmol/L及（7.39±4.16）nmol/L；蟾蜍灵能诱导肺癌细胞凋亡，形态学表现为出现凋亡小体及流式细胞仪检测到的亚二倍体凋亡峰，凋亡率与对照组比较差异有统计学意义（均*P* < 0.01）；蟾蜍灵诱导细胞凋亡过程中，下调Livin蛋白表达（*P* < 0.01），同时活化Caspase-3蛋白。

**结论:**

蟾蜍灵能够抑制肺癌细胞A549的增殖，并诱导其凋亡；抑制凋亡抑制蛋白Livin的活性及活化Caspase-3可能在其抑癌机制中发挥重要作用。

## Abstract (en)

**Background and objective:**

Bufalin, a component of the Chinese medicine chan'su, induces apoptosis in various human tumor cell lines. The aim of this study is to investigate the mechanism of anti-proliferation and the induction of apoptosis of Bufalin on non-small cell lung cancer cell.

**Methods:**

The effect of Bufalin on A549 cell proliferation was measured using MTT assay; the morphological change was observed with Wright-Giemsa stain; cell cycle phase distribution and hypodiploid DNA were determined by flow cytometry with PI; expressions of Livin, Caspase-3 were detected by Western blot.

**Results:**

MTT assay showed that Bufalin inhibited A549 cell proliferation in time and dose-dependent manner. The inhibition concentration of 50% cell growth (I_C50_) at 48 h, 72 h and 96 h were (56.14±6.72) nmol/L, (15.57±4.28) nmol/L and (7.39±4.16) nmol/L, respectively; apoptosis of A549 cells could be effectively induced by Bufalin; apoptotic bodies and sub-G_1_ peak (representing apoptosis) emerged when cells were treated with different concentrations, compared with the untreated control group (*P* < 0.01). The expression of Livin protein was downregulated (*P* < 0.01) and Caspase-3 protein was activated during Bufalin-induced apoptosis in A549 cells.

**Conclusion:**

Bufalin suppresses the growth of A549 cells and induces apoptosis; inhibition of Livin and activation of Caspase-3 may be involved in its mechanism.

非小细胞肺癌（non-small cell lung cancer, NSCLC）约占肺癌总数的80%-85%，而其中近1/3的患者初次确诊时已为局部晚期^[1]^，多数NSCLC患者可能在其病程的不同时期需要接受药物化疗。常用抗肿瘤药物的临床疗效有限，且抗瘤药物的诸多毒副作用如骨髓抑制、消化道反应等会严重影响肿瘤患者对化疗的耐受性和依从性。因此，寻找高效低毒的治疗药物成为近年来肿瘤基础和临床研究的热点。蟾蜍灵（Bufalin）是从中药蟾酥中提取出来的有效成分之一，体外实验和部分动物实验^[2, 3]^发现，蟾蜍灵可以选择性地诱导一系列不同来源的肿瘤细胞凋亡，但对正常宿主细胞无明显杀伤作用。在本实验中，我们研究了蟾蜍灵对NSCLC细胞株A549的诱导凋亡作用及其可能机制，现报道如下。

The article "Effect of Bufalin on Proliferation and Apoptosis of Human Non-small Cell Lung Cancer A549 Cell" was retracted in 2010. Reason: duplicate publication.

## 1 材料与方法

### 1.1 主要试剂

蟾蜍灵、碘化丙锭（propidium iodide, PI）、核糖核酸酶（ribonucleic acid enzyme, RNAse）、F12K培养基购于Sigma公司；胎牛血清购于中国医学科学院血液学研究所；兔抗人Caspase-3、β-actin抗体购于Santa Cruz公司；兔抗人Livin抗体购于博士德生物工程有限公司；羊抗兔辣根过氧化物酶标记的二抗购于北京中杉金桥生物技术有限公司；四甲基偶氮唑蓝（MTT）购于北京华美公司。将蟾蜍灵用无水乙醇配制成10 mmol/L的储存液，-20 oC贮存。实验前用磷酸盐缓冲液（phosphate-buffered saline, PBS）稀释，将乙醇终浓度控制在体积分数 < 0.01%。预实验表明，该浓度乙醇对细胞增殖无影响。

### 1.2 细胞培养

人肺腺癌细胞株A549购于中科院上海细胞库，置于含10%胎牛血清的F12K培养液中，37 ℃、5%CO_2_、饱和湿度的培养箱内传代培养，0.25%胰酶消化液消化传代，3天-4天传代1次。所有实验均采用对数生长期细胞。

### 1.3 MTT法进行细胞活力检测

取对数生长期细胞，常规胰酶消化制成单细胞悬液，将细胞浓度调至2×10^4^/mL-10×10^4^/mL接种于96孔板，每孔180 μL，培养过夜后分别加入终浓度为10 nmol/L、20 nmol/L、50 nmol/L、100 nmol/L和200 nmol/L的蟾蜍灵，空白组和对照组加入等量的培养液，每组设3个复孔，每孔终体积为200 μL。加药分别培养48 h、72 h和96 h，终止培养前4 h每孔加入MTT溶液（5 mg/mL）20 μL，到预定时间后吸去上清，每孔加入200 μL DMSO，振荡摇匀。用酶标仪于570 nm波长条件下测定吸光度。按下列公式计算细胞增殖抑制率: 增殖抑制率（%）=1-（处理组平均OD值-空白对照组平均OD值）/（对照组平均OD值-空白对照组平均OD值）×100%。计算蟾蜍灵抑制细胞增殖50%的药物浓度（IC_50_），并绘制细胞增殖抑制曲线。

### 1.4 瑞氏-吉姆萨染色法观察细胞形态变化

40 nmol/L蟾蜍灵作用细胞48 h后分别收集对照组及处理组细胞，2 000 r/min离心机甩片3 min制成细胞涂片，用瑞氏-吉姆萨染液染色，光学显微镜下观察细胞形态变化。

### 1.5 流式细胞术检测细胞周期分布及凋亡情况

用20 nmol/L、40 nmol/L、100 nmol/L蟾蜍灵分别作用细胞48 h、72 h，胰酶消化后收集细胞1 000 r/min离心5 min，冷PBS洗涤，加入70%的冷乙醇4 oC过夜，PBS再次离心洗涤，加入RNAse（10 μg/mL）37 oC孵育30 min后，加入终浓度为10 μg/mL的PI，避光反应30 min后使用流式细胞仪进行DNA含量测定，采用Cell Quest软件进行细胞各周期的百分比分析，同时判定凋亡细胞百分率。

### 1.6 Western blot方法检测Livin、Caspase-3蛋白表达水平

将对照组和蟾蜍灵作用后的细胞裂解于RIPA裂解液中，冰上裂解40 min后，12 000 r/min离心20 min，取上清，采用Lowry法进行蛋白定量。与3×样品缓冲液混合后煮沸5 min。将蛋白样品（50 μg/lane）在15%的SDS-聚丙烯凝胶中电泳约3 h，然后转印至硝酸纤维素膜上90 min。用5%脱脂奶粉封闭1 h后，按预染Marker标记的分子量剪裁转印膜，分别加入Livin抗体（1:300）、Caspase-3（1:1 000）抗体及β-actin抗体（1:1 000），过夜。TTBS洗4次后加入辣根过氧化物酶标记的二抗（1:800）作用30 min，ECL法显色后GIS凝胶图像分析系统拍照并分析处理。

### 1.7 统计学处理

所有数据均为3次独立实验结果，以Mean±SD表示，采用SPSS 13.0统计软件进行单因素方差分析和*t*检验。*P* < 0.05为差异有统计学意义。

## 2 结果

### 2.1 蟾蜍灵明显抑制A549细胞增殖

10 nmol/L-200 nmol/L蟾蜍灵分别作用A549细胞48 h、72 h及96 h，MTT结果显示，蟾蜍灵抑制细胞增殖呈时间、剂量依赖关系。48 h、72 h及96 h的IC_50_值分别为（56.14±6.72）nmol/L、（15.57±4.28）nmol/L及（7.39±4.16）nmol/L（图 1）。

**1:** 细胞增殖抑制曲线 The curve of cell proliferation inhibition

### 2.2 蟾蜍灵作用A549细胞后的形态学变化

用40 nmol/L蟾蜍灵作用A549细胞48 h后，瑞氏-吉姆萨染色，光镜下可以观察到细胞染色质固缩、胞核碎裂及凋亡小体形成等典型的凋亡细胞形态（图 2）。

**2:** 蟾蜍灵对A549细胞形态学的影响（瑞氏-吉姆萨染色，×400）。A：对照组；B：40 nmol/L。 The effect of Bufalin on A549 cell morphology (Wright-Giemsa, ×400). A: Control; B: 40 nmol/L.

### 2.3 蟾蜍灵诱导A549细胞凋亡

20 nmol/L、40 nmol/L、100 nmol/L蟾蜍灵分别作用细胞48 h及72 h后，流式细胞仪检测显示形成明显的亚二倍体凋亡峰（sub-G_1_峰），亚二倍体细胞百分数（细胞凋亡率）48 h分别为（2.93±0.67）%、（4.86±1.26）%及（7.34±1.85）%；72 h分别为（4.64±0.74）%、（9.86±1.63）%及（18.05±1.58）%，与对照组比较差异有统计学意义（均*P* < 0.01）（图 3），其余细胞周期分布无明显变化。

**3:** 流式细胞仪检测蟾蜍灵诱导的凋亡细胞。A：不同浓度蟾蜍灵培养A549细胞48 h及72 h；1：对照组（48 h）；2：20 nmol/L（48 h）；3：40 nmol/L（48 h）；4：100 nmol/L（48 h）；5：对照组（72 h）；6：20 nmol/L（72 h）；7：40 nmol/L（72 h）；8：100 nmol/L（72h）；B：蟾蜍灵诱导细胞凋亡（^*^：*P* < 0.01，与对照组比较）。 Analysis of apoptosis induced by Bufalin in A549 cells by flow cytometry. A: A549 cells were cultured 48 h and 72 h with different concentrations; 1: Control (48 h); 2: 20 nmol/L (48 h); 3: 40 nmol/L (48 h); 4: 100 nmol/L (48 h); 5: Control (72 h); 6: 20 nmol/L (72 h); 7: 40 nmol/L (72 h); 8: 100 nmol/L (72 h); B: Bufalin induces A549 cells apoptosis (Compared with control group, ^*^: *P* < 0.01).

The article "Effect of Bufalin on Proliferation and Apoptosis of Human Non-small Cell Lung Cancer A549 Cell" was retracted in 2010. Reason: duplicate publication.

### 2.4 蟾蜍灵对Livin蛋白表达的影响

用20 nmol/L、40 nmol/L、100 nmol/L蟾蜍灵分别作用细胞48 h，Western blot检测结果显示，Livin蛋白表达分别下调至作用前的（61.29±7.76）%、（29.03±4.63）%及（22.17±6.02）%，与对照组比较其差异具有统计学意义（均*P* < 0.01）（图 4）。

**4:** 蟾蜍灵对Livin蛋白表达的影响。1：对照组；2：20 nmol/L；3：40 nmol/L；4：100 nmol/L。 The expressions of Livin protein after treatment with Bufalin. 1: Control; 2: 20 nmol/L; 3: 40 nmol/L; 4: 100 nmol/L.

### 2.5 蟾蜍灵对Caspase-3蛋白活化的影响

Western blot结果显示，20 nmol/L蟾蜍灵作用细胞48 h仅检测到非活化状态32 kDa的Pro-Caspase-3，而40 nmol/L、100 nmol/L可检测到Caspase-3的活化亚基（17 kDa），且随浓度增大活化程度更明显（图 5）。

**5:** 蟾蜍灵对Caspase-3蛋白活化的影响。1：对照组；2：20 nmol/L；3：40 nmol/L；4：100 nmol/L。 The expressions of Caspase-3 protein after treatment with Bufalin. 1: Control; 2: 20 nmol/L; 3: 40 nmol/L; 4: 100 nmol/L.

## 3 讨论

蟾蜍灵是中药蟾酥的有效成分之一，国内外学者的研究报道，蟾蜍灵可以诱导部分白血病细胞及实体瘤细胞分化及凋亡。Amano等^[4]^研究表明蟾蜍灵可以通过增加维生素D_3_受体而增强1, 25(OH)_2_D_3_诱导髓样白血病细胞分化的能力，为进一步明确蟾蜍灵诱导白血病细胞分化提供了理论依据；Chen等^[5]^也通过基因表达图谱验证了蟾蜍灵诱导HL-60细胞凋亡过程中异常活化*NF-kB*及*AP-1*基因，但蟾蜍灵诱导细胞凋亡的确切机理尚未阐明，目前研究认为其作用机理与*survivin*、*c-myc*、*WT1*、*AP-1*等基因及MAPK信号通路调节相关。本研究结果显示蟾蜍灵可以时间、剂量依赖的方式抑制肺癌A549细胞增殖，同时诱导其凋亡。实验研究表明许多抗癌药物作用于肿瘤细胞，在低蟾蜍灵浓度、短时间时表现为周期阻滞，高浓度、长时间表现为凋亡。但目前关于蟾蜍灵引起细胞周期阻滞的报道不一，Li等^[6]^报道20 nmol/L蟾蜍灵作用胃癌MGC803细胞24 h后可引起明显的G_2_/M期阻滞；但Nasu等^[7]^报道蟾蜍灵引起子宫内膜异位基质细胞G_0_/G_1_期阻滞。在本研究中，流式细胞仪分析显示并未观察到明显的细胞周期阻滞，而是出现明显的亚二倍体凋亡峰，且经瑞氏-吉姆萨染色后亦可观察到处理组细胞染色质固缩、胞核碎裂及凋亡小体形成等典型的凋亡细胞形态。这些结果提示蟾蜍灵作用于不同的细胞系可能引起不同的细胞周期分布，其对细胞周期阻滞的影响可能存在细胞特异性。

凋亡抑制蛋白（inhibitor of apoptosis protein, IAP）家族是机体内抗凋亡因子之一，在肿瘤的形成过程中发挥着重要作用。Livin作为IAP家族的新成员，近年来研究表明，Livin的过度表达预示着肿瘤恶性度高、生存期短和预后不良，并可能是导致肿瘤细胞耐药的因素之一。在本实验中，蟾蜍灵诱导A549细胞凋亡过程中Livin蛋白的表达明显下调，相对应A549细胞的凋亡率随之上升。目前的许多研究^[8, 9]^已经通过把Livin作为靶点，在分子水平上抑制其表达而诱导肿瘤细胞凋亡并提高肿瘤细胞对促凋亡刺激的敏感性。

Caspases是一组天冬氨酸特异性的半胱氨酸蛋白酶，在细胞凋亡过程中起关键作用。Caspase-3是细胞凋亡的核心酶，被认为是细胞凋亡的中心环节和执行者。许多凋亡诱导剂可通过Caspase-3依赖的方式诱导肿瘤细胞凋亡。本实验结果显示，40 nmol/L、100 nmol/L蟾蜍灵作用A549细胞48 h可检测到Caspase-3（17 kDa）活化亚基，首次证实蟾蜍灵在诱导A549细胞凋亡过程中裂解活化Caspase-3，提示蟾蜍灵可通过Caspase-3依赖的方式诱导细胞凋亡。

目前研究^[10]^认为Livin主要是在蛋白水平通过BIR结构域与介导细胞凋亡的下游效应Caspases，即激活形式的Caspase-3和Caspase-7结合后抑制细胞凋亡。在Fas/Caspase-8诱导的死亡受体途径中，Livin直接抑制该途径中的核心酶Caspase-3发挥作用；而在另一条由细胞色素C（cytochrome c, Cyt-c）/凋亡蛋白活化因子1（apoptotic protease activating factor-1, Apaf-1）作用的线粒体途径中，Livin也能与Caspase-9的前体蛋白及其激活形式结合或通过阻断Caspase-3对Caspase-9前体蛋白的反馈激活从而产生抗凋亡的作用。在本实验中，蟾蜍灵作用A549细胞48 h后，随着药物浓度的增加，Livin蛋白的表达分别下调，而同时亦检测到Caspase-3蛋白的逐渐活化。由此可推测，蟾蜍灵作用肺癌A549细胞后，通过下调凋亡抑制蛋白Livin的表达，解除了IAP对Caspase-3的抑制，使Caspase-3蛋白裂解活化，即有活性的凋亡效应蛋白Caspase-3（17 kDa）表达上调，凋亡率随之增加，这同Livin具有抗凋亡作用的理论也是相吻合的。以上实验结果表明，一定浓度的蟾蜍灵在体外对人非小细胞肺癌A549细胞有显著的生长抑制作用，下调凋亡抑制蛋白Livin及活化Caspase-3是其诱导细胞凋亡机制之一，上述结果为蟾蜍灵进一步的实验研究提供了一定的理论依据，但其诱导细胞凋亡的确切机制有待今后进一步的研究来不断完善。
